# Seat Belt Aortic Dissection: A Case Report

**DOI:** 10.7759/cureus.4662

**Published:** 2019-05-14

**Authors:** Mohamed Ahmed, Ahmed Mahmoud, Michael Samotowka, Kristofer Mitchell, Rasha Saeed

**Affiliations:** 1 Surgery, University of California, Riverside, USA; 2 Surgery, Riverside Community Hospital, Riverside, USA; 3 Surgery, Memorial Hospital, Jacksonville, USA; 4 Surgery, St. Mark's Hospital, Salt Lake City, USA; 5 Surgery, Arrowhead Regional Medical Center, Fontana, USA

**Keywords:** aortic dissection, seat belt, motor vehicle accident

## Abstract

Eighteen-year-old restrained male driver involved in a flip over motor vehicle accident resulting in a seatbelt injury triad ( rectus abdominis muscle disruption, injury to the sigmoid colon and infra-renal aortic dissection). The patient did well after the surgical resection of the sigmoid colon, repair of the rectus abdominis muscle and endovascular repair of the aorta. Our objective is to shed light on this potentially fatal injury.

## Introduction

Seat-belt sign was described as a linear ecchymosis of the abdominal wall following a motor vehicle accident in 1962 by Garrett and Braunstein [1]. Hamilton in 1968 described seat-belt injuries (visceral and neck compression fracture) [2]. Recently, the uncommon triad of seatbelt-related abdominal wall disruption (AWD), hollow viscous injury, and distal abdominal aortic injury after a motor vehicle collision has been reported [3]. The increased use of seat belt over the last two decades led to a decrease in the motor vehicle accident-related mortality [4]. Direct compression of the aorta between the horizontal part of the seat belt and the vertebrae leads to dissection and thrombosis. We describe a case of seat belt injury triad.

## Case presentation

Eighteen-year-old restrained driver was brought to our emergency room after a flip over motor vehicle accident with back seat passenger fatality. Immediate intubation was done for a Glasgow coma scale of five. Focused assessment with sonography for trauma was negative. Bleeding scalp laceration repaired and left femur fracture splinted. He was admitted to the intensive care unit (ICU) after a pan scan concerning for filling defects (indeterminate intraluminal thrombi or dye mixing defects) within the infra-renal aorta extending into the bilateral common iliac artery (Figure 1) and a small subarachnoid hemorrhage.

**Figure 1:** Computed tomographic scan of the abdomen and pelvis. Filling defect in the aorta (Red arrow) indeterminant for clot or mixing of contrast defects

In spite of aggressive resuscitation, four hours after ICU admission, the patient continued to be acidotic ( lactic acid 4.3 mMol/L), tachycardic ( 120-130 beats per minutes), hypotensive (systolic blood pressure in the eighties) with a stable hemoglobin (12G/dl). The clinical picture was concerning for hallow viscous injury not apparent on initial computed tomographic (CT) scan as no other explanation for his worsening acidosis was found. Abdomen exploration with resection of de-vascularized sigmoid colon segment, ABTHERA (open abdomen negative pressure therapy) application with a planned return to the operating room the next day for re-exploration, colostomy diversion and repair of transected rectus abdominis muscle (Figure 2).

**Figure 2:** Abdomen re-exploration Transected rectus abdominis (blue arrow) Seat belt sign (red arrow) Transected sigmoid colon (black arrow)

Computed tomography angiography of the abdomen and pelvis with run off was obtained the day after due to loss of palpable pulses on both feet confirming infra-renal aortic injury (Figure 3).

**Figure 3:** Computed tomography angiography of abdomen and pelvis with run off Aortic dissection and clot (red arrow) Left common iliac clot (blue arrow)

Endovascular graft repair was determined to be a safer option given the patient subarachnoid hemorrhage treatment which limits the liberal use of anticoagulation needed in open aortic graft repair and his abdomen contamination by the sigmoid colon injury (Figure 4).

**Figure 4:** Complete angiogram after endovascular repair Stent (red arrow).

Patient femur fracture was initially managed with an external fixation device and intramedullary nail five days later. His general condition gradually improved and was discharged from the hospital to a rehabilitation facility after 20 days of admission with planned colostomy taken down eight weeks later.

## Discussion

Blunt traumatic AWD is increasingly recognized in adult trauma patients due to the liberal use of CT scan [5]. In contrast to AWD, blunt abdominal aortic injury is rare with estimated incidence up to 0.04% of non-penetrating trauma and only one-third were caused by seatbelt use [6-8]. Colon injury occurs in 1.1% of patients with blunt abdominal trauma [9]. CT imaging without oral contrast solution for blunt bowel and mesenteric injuries sensitivity (95% ) and specificity (99.6%) is a reason why abdomen exploration should be entertained in patients who continue to deteriorate in-spite of aggressive resuscitation and no other cause can be determined [10]. Early CT scan of the abdomen and pelvis is a common practice in trauma and delay in CT is associated with poor outcome in patients with blunt traumatic aortic injury [11]. Abnormal CT scan findings should always be followed up to avoid delay in diagnosis. Aortic blow-out rupture is a life-threatening and emergency laparotomy is required, however, partial aortic wall injury including dissection is a good indication for endovascular aortic repair (EVAR) [12-13]. EVAR is minimally invasive and preferred in the critically ill patient, when hollow viscous injury exist where open repair may carry a higher risk for graft infection, or when the liberal use of anticoagulation is contraindicated such as in our case of traumatic subarachnoid hemorrhage. In some cases it is difficult to ascertain the injury and intravascular ultrasound can be used to confirm the diagnosis of blunt abdominal aortic injury when CTA findings are equivocal [14]. 

## Conclusions

Blunt abdominal aortic injury (BAAI) is a significant life-threatening injury that should be considered in patients with significant trauma mechanism. Early diagnosis with CT improve patient outcomes. It may be associated with other organ injury and endovascular repair is a valuable minimally invasive option for critically ill patients. 

## References

[1] Wotherspoon S, Chu K, Brown A (2001). Abdominal injury and the seat‐belt sign. Emerg. Med.

[2] Hamilton J (1968). Seat-belt injuries. BMJ.

[3] Kulvatunyou N, Albrecht M, Bender J (2011). Seatbelt triad: severe abdominal wall disruption, hollow viscus injury, and major vascular injury. Am Surg.

[4] Al-Ozaibi L, Adnan J, Hassan B (2019). Seat belt syndrome: delayed or missed intestinal injuries, a case report and review of literature. Int J Surg Case Rep.

[5] Dennis R, Marshall A, Deshmukh H (2009). Abdominal wall injuries after blunt trauma: incidence and grading system. Am J Surg.

[6] Teruya T, Bianchi C, Abou-Zamzam A (2005). Endovascular treatment of a blunt traumatic abdominal aortic injury with a commercially available stent graft. Ann Vasc Surg.

[7] Voellinger D, Saddakni S, Melton S (2019). Endovascular repair of a traumatic infrarenal aortic transection: a case report and review. Vasc Surg.

[8] Fontaine A, Nicholls C, Borsa J (2019). Seat belt aorta: endovascular management with a stent-graft. JEVT.

[9] Katayama Y, Kitamura T, Hirose T (2019). Delay of computed tomography is associated with poor outcome in patients with blunt traumatic aortic injury: a nationwide observational study in Japan. Med.

[10] Allen T, Mueller M, Bonk R (2004). Computed tomographic scanning without oral contrast solution for blunt bowel and mesenteric injuries in abdominal trauma. J Trauma.

[11] Ricciardi R, Paterson C, Islam S (2004). Independent predictors of morbidity and mortality in blunt colon trauma. Am Surg.

[12] Gunn M, Campbell M, Hoffer E (2007). Traumatic abdominal aortic injury treated by endovascular stent placement. Emerg Radiol.

[13] ChenKaoa C, HaoHuang T, WeiChe C (2019). Blunt abdominal aortic injury may accompany bowel transection. Interact Cardiovas Thorac Surg.

[14] Shi Y, Tsai P, Wall M (2015). Intravascular ultrasound enhanced aortic sizing for endovascular treatment of blunt aortic injury. J Trauma Acute Care Surg.

